# DeepVariant-on-Spark: Small-Scale Genome Analysis Using a Cloud-Based Computing Framework

**DOI:** 10.1155/2020/7231205

**Published:** 2020-09-01

**Authors:** Po-Jung Huang, Jui-Huan Chang, Hou-Hsien Lin, Yu-Xuan Li, Chi-Ching Lee, Chung-Tsai Su, Yun-Lung Li, Ming-Tai Chang, Sid Weng, Wei-Hung Cheng, Cheng-Hsun Chiu, Petrus Tang

**Affiliations:** ^1^Department of Biomedical Sciences, Chang Gung University, Taoyuan, Taiwan; ^2^Graduate Institute of Biomedical Sciences, College of Medicine, Chang Gung University, Taoyuan, Taiwan; ^3^Genomic Medicine Core Laboratory, Chang Gung Memorial Hospital, Linkou, Taiwan; ^4^Institute of Bioinformatics and Structural Biology, National Tsing Hua University, Hsinchu, Taiwan; ^5^Department of Computer Science and Information Engineering, Chang Gung University, Taoyuan, Taiwan; ^6^ATGENOMIX INC, Rm. 918, 9F, 96, Chia Hsin Bldg. (Second Bldg.) Sec. 2, Zhongshan N. Rd., Zhongshan Dist., Taipei, Taiwan; ^7^Department of Parasitology, College of Medicine, Chang Gung University, Taoyuan, Taiwan

## Abstract

Although sequencing a human genome has become affordable, identifying genetic variants from whole-genome sequence data is still a hurdle for researchers without adequate computing equipment or bioinformatics support. GATK is a gold standard method for the identification of genetic variants and has been widely used in genome projects and population genetic studies for many years. This was until the Google Brain team developed a new method, DeepVariant, which utilizes deep neural networks to construct an image classification model to identify genetic variants. However, the superior accuracy of DeepVariant comes at the cost of computational intensity, largely constraining its applications. Accordingly, we present DeepVariant-on-Spark to optimize resource allocation, enable multi-GPU support, and accelerate the processing of the DeepVariant pipeline. To make DeepVariant-on-Spark more accessible to everyone, we have deployed the DeepVariant-on-Spark to the Google Cloud Platform (GCP). Users can deploy DeepVariant-on-Spark on the GCP following our instruction within 20 minutes and start to analyze at least ten whole-genome sequencing datasets using free credits provided by the GCP. DeepVaraint-on-Spark is freely available for small-scale genome analysis using a cloud-based computing framework, which is suitable for pilot testing or preliminary study, while reserving the flexibility and scalability for large-scale sequencing projects.

## 1. Introduction

As the cost of sequencing a human genome decreased dramatically, large-scale whole-genome sequencing projects were launched alongside the rising demand for precision medicine. Previous studies have stated that interethnic differences in drug response are substantial, and precision medicine relies on genotype-based prescribing decisions aimed at mitigating the risks and maximizing the efficacy of pharmacotherapy. Accordingly, national projects, such as those in the UK, United States, EU, Mexico, India, China, Sweden, Korea, and Taiwan biobank [1–8], have been launched and exemplify this trend.

To the best of our knowledge, the GATK [9–11] is one of the dominant packages for the identification of germline genetic variants and has been widely used in genome projects [12–15] and applied to the analyses of 125,748 exomes and 15,708 genomes (https://gnomad.broadinstitute.org/about) as part of population genetic studies. In 2016, the Google Brain team announced DeepVariant [16], which utilizes deep neural networks to construct an image classification model to identify genetic variants. DeepVariant outperforms GATK—a golden standard method for variant calling—and has won the PrecisionFDA Truth Challenge Award for the highest SNP performance. Supernat et al. have confirmed the results of the PrecisionFDA Truth Challenge, proving that DeepVariant is currently the most precise variant caller available [16].

DeepVariant's superior accuracy comes at the cost of computational intensity, as it requires approximately two times longer wall-clock times than GATK in variant identification. DeepVariant is composed of three steps: (1) make_examples obtains BAM files and converts them to images, (2) call_variants performs the variant calling using the ML-trained model, and (3) post process_variants transforms the variant calling output into a standard VCF file. Following the authors' instructions, call_variants is the only step that can make use of GPUs to reduce the variant calling time by more than 50% [16]. However, overcoming the configuration hurdle of GPU hardware can be difficult for users without bioinformatics experience. Furthermore, the call_variants step currently only supports one GPU, and the other two steps of DeepVariant are not optimized for speed, indicating that there is room for improvement.

Our specific aim in constructing DeepVariant-on-Spark is to enable multi-GPU support and optimize resource allocation in the DeepVariant pipeline. DeepVaraint-on-Spark leverages the Apache Spark and Hadoop technologies to launch DeepVariant processes in parallel and ensure that we can fully utilize all GPU resources. To make DeepVariant-on-Spark more accessible to everyone, we have deployed DeepVariant-on-Spark onto the Google Cloud Platform (GCP). Users can follow our step-by-step instruction, and all necessary packages can be installed automatically by Ansible [17] within 20 minutes. DeepVariant-on-Spark can analyze at least ten whole-genome sequencing tasks using the 300 free USD credits provided by the GCP, which is suitable for preliminary studies or pilot testing. On the other hand, DeepVariant-on-Spark also provides the flexibility and scalability for large-scale sequencing projects.

## 2. Materials and Methods

### 2.1. Deployment of DeepVariant-on-Spark

DeepVariant-on-Spark is designed as a cloud-based application, utilizing Google Cloud Dataproc (https://cloud.google.com/dataproc/) to manage services for running Apache Spark [18] and Hadoop [19] clusters in a fast, more straightforward, and efficient way. Installing the gsutil tool is the first step and enables users to access the Google Cloud Dataproc and publicly accessible objects (https://cloud.google.com/storage/docs/gsutil_install). Cloud Dataproc provides a mechanism for automating cluster resource management, which enables flexible addition and subtraction of cluster nodes. After successfully launching the DataProc cluster, Ansible is used to automate the deployment of all necessary packages to the entire cluster, which includes DeepVariant [20], Adam [21], SeqPiper, and PiedPiper, using the YAML language in the form of Ansible playbooks. Detailed installation instructions can be found on the tutorial page (https://storage.cloud.google.com/sparkdv/performance-test/DeepVariant-On-Spark_Tutorial.html?hl=zh-TW).

### 2.2. Whole-Genome Sequencing and Alignment of the NA12878 Reference Sample

The 30x whole-genome sequencing of the NA12878 reference sample was downloaded from the European Nucleotide Archive (ENA), which was sequenced by an Illumina NovaSeq 6000 instrument with a 150 bp paired-end sequencing protocol. Reads were aligned to the human reference genome—Gencode GRCh38.p13 by bwa-mem. We deposited the aligned sequences in Google Storage as a BAM file (gs://sparkdv/performance-test/NA12878-novaseq.bam) and used Qualimap2 to evaluate the alignment quality of the obtained BAM file [22].

### 2.3. Framework of DeepVariant-on-Spark

Currently, DeepVariant only supports single GPU acceleration in variant calling, and we cannot obtain any benefit on machines with multiple GPUs. Therefore, DeepVariant-on-Spark was designed to leverage Apache Spark to launch multiple DeepVariant processes in parallel to address the scalability problem of variant calling. The input BAM file was first uploaded to the Hadoop Distributed File System (HDFS), followed by segmentation into several 1 Mbp data blocks. Then, we transformed the resulting data blocks into Apache Parquet file format (∗.parquet) to enhance the transfer performance through data compression. To overcome the load imbalance introduced by the uneven length of chromosomes, we aggregated those 1 Mbp data blocks into 155 approximately equal-sized BAM files according to contiguous unmasked regions of the human genome. These BAM files were transformed into resilient distributed datasets (RDD) data structure, which can be further partitioned and distributed across a Spark cluster. Finally, the Spark PipeRDD was used to parallelize the DeepVariant processes on Spark to ensure that all the GPU resources can be fully utilized across compute nodes (Figure 1).

### 2.4. Quality Evaluation of Variant Calling

We performed variant calling using DeepVariant and DeepVariant-on-Spark to obtain variant call format (VCF) files from the NA12878 reference sample. DeepVariant version 0.7.0 was used for constructing the original DeepVariant pipeline and our accelerated DeepVariant-on-Spark pipeline on the cloud computing environment. The results from both pipelines with different CPU/GPU combinations were compared to the GIAB NIST v3.2.2 HG001 truth data [23, 24] (ftp://ftp-trace.ncbi.nlm.nih.gov/giab/ftp/release/NA12878_HG001/NISTv3.3.2/GRCh38/) to determine the *F*-score, recall, and precision values for SNPs and Indels. The RTG vcfeval tool (https://github.com/RealTimeGenomics/rtg-tools) was used to generate intermediate VCF for variant comparison [25]. Illumina's hap.py (https://github.com/Illumina/hap.py/blob/master/doc/happy.md), a quantify tool, was utilized to count and stratify variants.

### 2.5. Data Access

The DeepVariant v0.7.0 used in this study is available on the following GitHub page: https://github.com/google/deepvariant/releases/tag/v0.7.0.

The DeepVariant-on-Spark pipeline used in this study is available on the following GitHub page: https://github.com/atgenomix/deepvariant-on-spark.

The GIAB NIST v3.3.2 true variant dataset used for evaluating variant caller performance can be downloaded through the following link: ftp://ftp-trace.ncbi.nlm.nih.gov/giab/ftp/release/NA12878_HG001/NISTv3.3.2/GRCh38/.

Variant evaluation and comparison tools can be obtained from https://github.com/RealTimeGenomics/rtg-tools and https://github.com/Illumina/hap.py.

## 3. Results

### 3.1. Comparison of the DeepVariant and DeepVariant-on-Spark for Analysis of Human 30x WGS Data

First, we need to confirm that DeepVariant-on-Spark can achieve comparable accuracy to DeepVariant. Before we can perform a side-by-side comparison between DeepVariant-on-Spark and DeepVariant, we need to have a standard BAM file for the evaluation of the variant calling accuracy. The 30x WGS of the NA12878 reference sample with 611,997,146 reads was aligned to the GRCh38.p13 reference genome to obtain the BAM file, with 99.82% aligned reads, 41.25% GC, and 29.08x mean coverage. Our analysis showed that the *F*-scores, the harmonic mean of the recall, and precision, for both SNVs and Indels, were the same (*F*-scores of 0.99940 and 0.96168, respectively) for DeepVariant-on-Spark as compared to DeepVariant. As shown in Table 1, the analyses have been comprehensively performed under different combinations of hardware settings, and the results were consistent.

### 3.2. The Computation Bottlenecks of DeepVariant

To explore the bottleneck of DeepVariant, we evaluated the DeepVariant pipeline on the GCP using a virtual machine equipped with 16 CPUs (2.0 GHz) and 60 GB of memory, with flexibility for adding or removing CPU/GPU on existing virtual machine instances. The reference runtime for DeepVariant was established using 16 CPUs (2.0 GHz), which took 17.5 hours to finish variant calling from 30x WGS. The results show that “Make_Examples” and “Call_Variants” are computational bottlenecks of the DeepVariant pipeline. Increasing the number of CPUs may have improved both steps, but the impact on the “Call_Variants” step is not apparent (Figure 2(a)). However, when the number of CPUs increases, DeepVariant-on-Spark can provide a significant improvement in both the “Make_Examples” and “Call_Variants” steps, resulting in an ideal speedup ratio for the overall processes (Figures 2(a) and 2(b)). Only two compute nodes, which are equivalent to 32 CPUs, are required by DeepVariant-on-Spark to achieve the same computing performance as DeepVariant with 64 CPUs. In addition, the GCP has limited the maximum number of CPUs for a single virtual machine to 96, leading to poor scalability of DeepVariant. We present DeepVariant-on-Spark with a scalable architecture for parallel execution of DeepVariant based on the Apache Spark framework. The distributed Apache Spark framework provides an excellent solution for addressing this scalability issue. DeepVariant-on-Spark can accelerate the default DeepVariant pipeline by seven times, taking the full load of 128 CPUs through 8 compute nodes, thereby achieving high performance due to the memory-based computing and good scalability on multiple nodes. We can reduce the overall wall-clock time for the variant calling of 30x WGS from 17.5 to 2.5 hours using 128 CPUs under the DeepVariant-on-Spark frameworks.

### 3.3. Scalability Analysis of DeepVariant and DeepVariant-on-Spark Based on Heterogeneous Computing Architecture

Heterogeneous computing, which uses a different type of processor (CPU or GPU) to gain efficiency and performance, therein incorporating specialized processing capabilities to handle specific tasks, has been gaining popularity in the past few years. Accordingly, we attempted to incorporate GPUs into existing virtual machine instances on the GCP. The results show that GPU acceleration is trivial at the “Make_Examples” step, whereas it introduces significant improvements at the “Call_Variants” step. The speedup rate increases after incorporating the GPUs (Figures 2(b) and 2(d)); however, we cannot find additional benefit from multiple GPUs, indicating that the current release of the DeepVariant pipeline supports a single GPU (Figure 2(b)). Accordingly, we introduce DeepVariant-on-Spark to unleash the full power of multiple GPUs. DeepVariant-on-Spark is evaluated on Google Cloud DataProc Spark clusters with 2, 4, and 8 compute nodes (Figures 2(c) and 2(d)). Each node is equipped with 16 CPUs (2.0 GHz), 104 GB of memory, and 1 NVIDIA Tesla P100 GPU processor. Through DeepVariant-on-Spark, not only the CPUs but also all the GPU resources can be fully utilized across multiple nodes, and we can reduce the wall-clock times for the “Call_Variants” step by ~45% when we double the number of GPUs. With eight compute nodes, which is equivalent to 128 CPUs and 8 NVIDIA Tesla P100 GPU processors, we can reduce the overall wall-clock time from 17.5 to 1.51 hours for the variant calling of 30x WGS. As shown in Figure 2(d), when we use 128 CPUs and 8 GPUs, we can accelerate the pipeline by 11 times, and the speedup ratio is still increasing, indicating that DeepVariant-on-Spark can achieve a high CPU and GPU utilization rate and is more scalable than the original DeepVariant pipeline.  Table 2 describes the wall-clock times of DeepVariant-on-Spark and DeepVariant with 1, 2, 4, and 8 compute nodes equipped with different CPU and GPU processors.

### 3.4. The Cost Effectiveness and Cost Efficiency of DeepVariant and DeepVariant-on-Spark

The primary purpose of this study is to provide a reference guide for users who plan to initiate a small-scale genome analysis to select their ideal solutions for their preliminary study. When computing time is not a major concern, the original DeepVariant pipeline with 16 CPUs can be a relatively cost-effective solution, which can analyze as many as 21 WGS datasets within the 300 USD free credits provided by the GCP. However, the default virtual machine architecture provided by the GCP has poor scalability, with a constraint on CPU number, making it difficult to optimize the trade-offs between cost and performance in running DeepVariant. At the same cost of 25 USD, DeepVariant takes 5.5 hours to finish a 30x WGS variant calling task with its inherited constraint of using 96 CPUs, while DeepVariant-on-Spark has the flexibility to adjust the cost-performance ratio to finish the same task in 2.5 hours. If pressed for time, DeepVariant-on-Spark would be a cost-efficient option that can finish the variant calling of 10 WGS data in just one day.  Table 2 summarizes the wall-clock times and cost estimates for analyzing 30x WGS on the GCP.

## 4. Discussion

In this study, we provide a flexible and scalable framework for DeepVariant acceleration. DeepVariant is the most precise variant caller that outperforms existing tools in SNV and Indel identification, therein having great potential for implementation in routine genetic diagnosis. Our proposed framework, DeepVariant-on-Spark, can not only reduce the wall-clock time while maintaining the same accuracy but also break the limitation on the number of utilizable CPUs and GPUs of DeepVariant.

The user needs to set up a new account on the GCP to receive the free credits, which can provide a convenient place to run DeepVariant with CPU and GPU support. Following the author's instructions, we can easily set up the CPU version of DeepVariant without any hurdles. However, we have to recompile a compatible NVIDIA GPU driver for a specific DeepVariant version on the GCP to enable the support of GPU hardware, which can be a challenge for inexperienced users. On the other hand, DeepVaraint-on-Spark provides step-by-step instructions on how to prepare a Google DataProc cluster. The installation script will recognize the hardware specifications and automatically deploy related drivers and packages to enable CPU or GPU acceleration of DeepVariant-on-Spark within 20 minutes. To the best of our knowledge, substantial efforts, such as Nextflow, DNAnexus, DNAstack, and Parabricks, have been devoted to accelerating the DeepVariant pipeline. Nextflow offers parallel processing of multiple samples for DeepVariant at a time [26], producing the results in a convenient and reproducible manner; however, the total wall-clock time for each sample is unchanged. DNAnexus and DNAstack can provide parallelized execution of DeepVariant with a GUI interface, but licenses are required to obtain the full functionality of these commercial packages. Parabricks introduced an accelerated DeepVaraint pipeline with multi-GPU support. However, license fees will be charged for all attached GPUs to receive their maximum performance. Google Genomics also suggests a cost-optimized configuration, using 32 virtual machines with 16 CPUs and 32 virtual machines with 32 CPUs for the “Make_Examples” and “Call_Variants” step, respectively, to complete the DeepVariant pipeline for 30x whole genome sample in 1 to 2 hours at a cost of between 3 USD and 4 USD. The configuration takes advance of CPUs from preemptible virtual machines, which are 80% cheaper than regular virtual machines. However, the compute engines might terminate at any time without guaranteeing turnaround time and are recommended only for fault-tolerant applications and users familiar with the GCP. Furthermore, a billable account is required to launch the preemptible virtual machines, and free credits for new users are not allowed for the acquisition of compute resources. Unlike most of the solutions mentioned above, DeepVariant-on-Spark is free for academic use. Despite not being the most cost-optimized solution available, DeepVariant-on-Spark can complete variant calling for 30x whole genome sample in 1.51 hours, which is comparable with the cost-optimized solution provided by Google Genomics. The reduction in wall-clock time to process a single 30X WGS sample is crucial in clinical settings where a result is needed to quickly take a diagnostic decision. When we were preparing this manuscript, multi-GPU support has been implemented in the recent release of DeepVaraint, making some of the benefits of DeepVariant-on-Spark become redundant. However, DeepVariant-on-Spark supports multi-GPU across multiple nodes, which seems to be conceptually better than limited to a single node.

To conclude, we present DeepVariant-on-Spark, a flexible and scalable tool for variant calling based on the Spark framework. DeepVariant-on-Spark implements the parallelization of the DeepVariant algorithm on a multinode cluster and enables the support of multiple GPUs, therein accelerating the processing of the DeepVariant pipeline while maintaining accuracy. Following our instructions, users can easily deploy the DeepVariant-on-Spark on the GCP within 20 minutes and start to analyze WGS datasets on the GCP, which is also useful for researchers who plan to initiate a small-scale genome analysis for preliminary study and makes DeepVariant, the TensorFlow-based variant caller, more attractive to general users, simplifying the usage to catalyze DeepVairant to a more broadly used tool.

## Figures and Tables

**Figure 1:** Framework of DeepVaraint-on-Spark. DeepVariant-on-Spark is based on the Google Dataproc service. After importing the BAM file into the DeepVariant-on-Spark cluster, the BAM file will be segmented into several 1 Mbp blocks in the “Adam Transform” step, and these blocks will be merged into 155 small BAM files in the “Select BAM” step. The 1 Mbp blocks and small BAM files are stored in the HDFS. PiedPiper will pipe the path of each BAM file to SeqPiper, which launches DeepVariant to produce the VCF file. Finally, in the “Merge VCFs” steps, each VCF file will be merged into a complete VCF file.

**Figure 2:** Wall-clock time and speedup of DeepVariant and DeepVariant-on-Spark with different combinations of CPU/GPU. Runtime comparison of DeepVariant and DeepVariant-on-Spark with different combinations of CPU/GPU. (a) DeepVariant runs on the pure CPU machine. (b) DeepVariant runs on the CPU/GPU hybrid machine. (c) DeepVariant-on-Spark runs on the pure CPU cluster. (d) DeepVariant-on-Spark runs on the CPU/GPU hybrid cluster. AdamTransform, SelectBAM, Make_Examples, Call_Variants, Postprocess_Variants, and Merge VCF represent each step in DeepVariant or DeepVariant-on-Spark. Speedup represents how many times each condition is faster than DeepVariant's (16 CPU) mode. The speed improvement of DeepVariant-on-Spark over DeepVariant is provided above. DeepVariant-on-Spark using 128-CPU and 8-GPU configurations improved the wall-clock time by 11.58x compared to DeepVariant using 16 CPUs.

**Table 1:** Comparison of variant calling results of DeepVariant and DeepVariant-on-Spark with different combinations of CPUs/GPUs.

Variant calling pipeline	Variant type	CPU^a^	GPU^b^	F1^c^	Recall	Precision	True positive	False negative	False positive	Genotype mismatch	Total number of SNV calls
DeepVariant	SNP	16	0	0.99940	0.99937	0.99943	3040855	1928	1744	363	3886287
		32	0	0.99940	0.99937	0.99943	3040856	1927	1744	363	3886337
		64	0	0.99940	0.99937	0.99943	3040856	1927	1744	363	3886366
		96	0	0.99940	0.99937	0.99943	3040855	1928	1744	363	3886339
		16	1	0.99940	0.99937	0.99943	3040855	1928	1744	363	3886287
		16	4	0.99940	0.99937	0.99943	3040855	1928	1744	363	3886287
		32	2	0.99940	0.99937	0.99943	3040856	1927	1744	363	3886337
		64	4	0.99940	0.99937	0.99943	3040856	1927	1744	363	3886366
DeepVariant-on-Spark		32	0	0.99940	0.99937	0.99943	3040856	1927	1744	363	3886403
		64	0	0.99940	0.99937	0.99943	3040856	1927	1744	363	3886403
		128	0	0.99940	0.99937	0.99943	3040856	1927	1744	363	3886403
		32	2	0.99940	0.99937	0.99943	3040856	1927	1744	363	3886403
		64	4	0.99940	0.99937	0.99943	3040856	1927	1744	363	3886404
		128	8	0.99940	0.99937	0.99943	3040856	1927	1744	363	3886403

DeepVariant	Indel	16	0	0.96168	0.95711	0.96628	478265	21432	17373	11151	868527
		32	0	0.96168	0.95711	0.96628	478265	21432	17373	11151	868535
		64	0	0.96168	0.95711	0.96628	478265	21432	17373	11151	868520
		96	0	0.96168	0.95711	0.96628	478265	21432	17373	11151	868535
		16	1	0.96168	0.95711	0.96628	478265	21432	17373	11151	868527
		16	4	0.96168	0.95711	0.96628	478265	21432	17373	11151	868528
		32	2	0.96168	0.95711	0.96628	478265	21432	17373	11151	868535
		64	4	0.96168	0.95711	0.96628	478265	21432	17373	11151	868520
DeepVariant-on-Spark		32	0	0.96168	0.95711	0.96628	478265	21432	17373	11151	868541
		64	0	0.96168	0.95711	0.96628	478265	21432	17373	11151	868541
		128	0	0.96168	0.95711	0.96628	478265	21432	17373	11151	868541
		32	2	0.96168	0.95711	0.96628	478265	21432	17373	11151	868542
		64	4	0.96168	0.95711	0.96628	478265	21432	17373	11151	868542
		128	8	0.96168	0.95711	0.96628	478265	21432	17373	11151	868541

^a^CPU means the number of CPU cores. ^b^GPU means the number of NVIDIA Tesla P100 GPUs. ^c^F1 means F1 score calculated by 2∗(recall∗precision)/(recall + precision).

**Table 2:** Comparison of the wall-clock time of DeepVariant and DeepVariant-on-Spark with different combinations of CPUs/GPUs.

Variant caller	DeepVariant							DeepVariant-on-Spark					
Machine model	CPU only				CPU+GPU			CPU only			CPU+GPU		
CPU^a^	16	32	64	96	16	32	64	32	64	128	32	64	128
GPU^b^	0	0	0	0	1	2	4	0	0	0	2	4	8
Spark^c^	No	No	No	No	No	No	No	Yes	Yes	Yes	Yes	Yes	Yes
AdamTransform (hr)	0	0	0	0	0	0	0	0.56	0.32	0.2	0.58	0.31	0.2
SelectBAM (hr)	0	0	0	0	0	0	0	0.5	0.33	0.23	0.48	0.29	0.2
Make_examples (hr)	6.13	3.15	1.73	1.2	5.93	3.1	1.6	2.72	1.6	1	2.82	1.48	0.83
Call_variants (hr)	10.8	6.53	5.35	3.83	1.51	1.52	1.5	3.66	2.02	0.98	0.7	0.38	0.21
Postprocess_variants (hr)	0.56	0.54	0.53	0.48	0.46	0.46	0.45	0.2	0.13	0.07	0.2	0.1	0.06
Merge VCF (hr)	0	0	0	0	0	0	0	0.02	0.02	0.02	0.02	0.02	0.02
Total time (hr)	17.49	10.22	7.61	5.51	7.9	5.08	3.55	7.66	4.42	2.5	4.8	2.58	1.52
USD/per genome	14.02	15.94	20.77	25.31	17.86	22.72	31.76	23.25	23.98	25.54	28.57	29.23	33.17
#genomes/300USD^d^	21	18	14	11	16	13	9	12	12	11	10	10	9

^a^CPU means the number of CPU cores. ^b^GPU means the number of NVIDIA Tesla P100 GPU. ^c^Spark means using Apache Spark or not. ^d^#genomes/300USD means the numbers of whole-genome sequence jobs that can be completed under the trial credit of 300 USD.

## Data Availability

The authors declare that the data supporting the findings of this study are available within the article.
